# At What Level of Heat Load Are Age-Related Impairments in the Ability to Dissipate Heat Evident in Females?

**DOI:** 10.1371/journal.pone.0119079

**Published:** 2015-03-19

**Authors:** Jill M. Stapleton, Martin P. Poirier, Andreas D. Flouris, Pierre Boulay, Ronald J. Sigal, Janine Malcolm, Glen P. Kenny

**Affiliations:** 1 Human and Environmental Physiology Research Unit, University of Ottawa, Ottawa, Ontario, Canada; 2 FAME Laboratory, Department of Exercise Science, University of Thessaly, Trikala, Greece; 3 Faculty of Physical Activity Sciences, University of Sherbrooke, Sherbrooke, Quebec, Canada; 4 Departments of Medicine, Cardiac Sciences and Community Health Sciences, Faculties of Medicine and Kinesiology, University of Calgary, Calgary, Alberta; 5 The Division of Endocrinology and Metabolism, Ottawa Hospital—Riverside Campus, Ottawa, Ontario, Canada; 6 Clinical Epidemiology Program, Ottawa Hospital Research Institute, Ottawa, Ontario, Canada; Louisiana State University, UNITED STATES

## Abstract

Studies have reported that older females have impaired heat loss responses during work in the heat compared to young females. However, it remains unclear at what level of heat stress these differences occur. Therefore, we examined whole-body heat loss [evaporative (H_E_) and dry heat loss, via direct calorimetry] and changes in body heat storage (∆H_b_, via direct and indirect calorimetry) in 10 young (23±4 years) and 10 older (58±5 years) females matched for body surface area and aerobic fitness (VO_2_peak) during three 30-min exercise bouts performed at incremental rates of metabolic heat production of 250 (Ex1), 325 (Ex2) and 400 (Ex3) W in the heat (40°C, 15% relative humidity). Exercise bouts were separated by 15 min of recovery. Since dry heat gain was similar between young and older females during exercise (p=0.52) and recovery (p=0.42), differences in whole-body heat loss were solely due to H_E_. Our results show that older females had a significantly lower H_E_ at the end of Ex2 (young: 383±34 W; older: 343±39 W, p=0.04) and Ex3 (young: 437±36 W; older: 389±29 W, p=0.008), however no difference was measured at the end of Ex1 (p=0.24). Also, the magnitude of difference in the maximal level of H_E_ achieved between the young and older females became greater with increasing heat loads (Ex1=10.2%, Ex2=11.6% and Ex3=12.4%). Furthermore, a significantly greater ∆H_b_ was measured for all heat loads for the older females (Ex1: 178±44 kJ; Ex2: 151±38 kJ; Ex3: 216±25 kJ, p=0.002) relative to the younger females (Ex1: 127±35 kJ; Ex2: 96±45 kJ; Ex3: 146±46 kJ). In contrast, no differences in H_E_ or ∆H_b_ were observed during recovery (p>0.05). We show that older habitually active females have an impaired capacity to dissipate heat compared to young females during exercise-induced heat loads of ≥325 W when performed in the heat.

## Introduction

A number of studies have shown that thermoregulatory function (i.e., heat loss through sweating and skin blood flow) during exercise is compromised in older compared to younger males [1,2,3,4,5,6,7]. However, there have been very few studies that have examined the effects of aging on the body’s ability to dissipate heat during exercise in females [8,9,10,11], all of which showed that older females have impaired tolerance to work in the heat. While these studies consistently demonstrated that aging in females is associated with impairments in heat dissipation, it remains unclear if the impairment in heat loss only occurs above a certain level of heat load (defined as the sum of metabolic heat production and dry heat exchange) and therefore requirement for heat loss.

At the onset of dynamic exercise, there is an instant and rapid elevation in the rate of metabolic heat production. However, this immediate increase in heat production is not initially offset by an increase in the rate of whole-body heat loss. Thus, the thermal imbalance caused by the lag in the activation of thermoefferent activity (i.e., sweating and skin blood flow) relative to the rapid gain in heat production causes pronounced increases in body heat storage during the early stages of exercise. A decrease in thermosensitivity and/or delay in the onset threshold, as previously shown to occur in older adults [5,6,12,13], would increase the duration of this heat imbalance resulting in a greater amount of heat stored in the body. This is consistent with a recent study by Larose *et al*. [8] who observed marked reductions in whole-body evaporative heat loss in older compared to young females after the first 10 min of exercise. This resulted in greater heat storage during four short intermittent (i.e., 15 min) exercise bouts performed at a fixed rate of metabolic heat production of 300 W [equivalent to ~44% peak oxygen uptake (VO_2_peak)] in the heat [35°C and 20% relative humidity (RH)] [8].

While the aforementioned study by Larose *et al*. [8] demonstrated age-related differences in the body’s physiological ability to dissipate heat occurs in the early stages of exercise during a moderate heat load (metabolic plus environmental heat load equivalent to ~320 W), it was not possible to discern if these age-related differences are observed with extended periods of exercise. As such, it is unknown if older females are able to achieve heat balance (i.e., rate of heat production matched with rate of heat loss), and therefore a stable core temperature, as exercise continues. A sustained reduction in whole-body heat loss would result in a progressive increase in body heat storage. If left unchecked, this could result in a heat-related injury or even death. In fact, previous studies reported that older females demonstrate attenuated local sweat rates as early as 30-min during a 2-h exercise protocol (35–40% VO_2_peak) in a hot, dry environment (48°C, 10% RH) compared to younger females matched for aerobic fitness, body surface area, and body adiposity [9,11]. A reduction in the level of sudomotor activity achieved for a given heat load, and therefore requirement for heat loss, would result in a greater heat storage and core temperature response as observed in these previous studies [9,11]. While these findings provide some evidence to suggest that age-related impairments are sustained with prolonged exercise, it remains unclear if age-related differences in the physiological capacity to dissipate heat remain intact or increase as the heat load becomes greater.

In light of the above knowledge gaps, the purpose of this study was to determine if age-related differences in whole-body heat loss are only evidenced above a certain heat load, and therefore requirement for heat loss, and if the degree of impairment augments with increases in heat load. To achieve this objective, we compared whole-body heat loss as assessed using direct calorimetry in young and older females during three 30-min intermittent exercise bouts performed at increasing levels of metabolic heat production of 250, 325 and 400 W, each separated by 15-min of recovery, under a constant environmental heat load (40°C and 15% RH). These rates of metabolic heat production were chosen to ensure that a compensable heat stress condition was achieved during the first exercise bout, progressing to a fully uncompensable condition during the final exercise bout for the older females. Based on previous studies showing differences in heat loss between young and older females at moderate levels of heat load (i.e., ~320 W or ~40% VO_2_peak), we hypothesized that differences in the capacity to dissipate heat between young and older females would occur at or near this threshold and that the magnitude of difference would become greater with progressive increases in heat load. As a consequence, older females would increasingly store more heat with elevated levels of heat stress.

## Methodology

### Ethics statement

The experimental protocol was approved by the University of Ottawa Health Sciences and Science Research Ethics Board, in accordance with the Declaration of Helsinki. Volunteers provided written informed consent before participating in the study.

### Participants

Twenty females volunteered for the study and were divided into two groups of 10 young (23 ± 4 years) and 10 older (58 ± 5 years) females. Participants were matched for height (young: 1.66 ± 0.02 m; older: 1.66 ± 0.04 m, p = 0.73), body mass (young: 63.6 ± 5.9 kg; older: 60.0 ± 4.9 kg, p = 0.16), body surface area (young: 1.70 ± 0.07 m^2^; older: 1.67 ± 0.08 m^2^, p = 0.23), body fat percentage (young: 23.9 ± 5.2%; older: 24.3 ± 5.7%, p = 0.76) and VO_2_peak (young: 39.7 ± 8.0 mLO_2_·kg^-1^·min^-1^; older: 39.0 ± 7.7 mLO_2_·kg^-1^·min^-1^, p = 0.80). All participants were non-smokers and did not report any history of hypertension, heart disease, diabetes or autonomic disorders. The young female participants had not taken medications except monophasic oral contraceptive, which provided 30–35 μg of ethinyl estrogen and low dose progestin for 21 days and placebo for 7 days. To control for hormonal effects, the younger females were tested in the early to mid-follicular phase (1–9 days after the onset of menstruation). All older females were postmenopausal; however two of the older females were on hormone replacement therapy. A 3-month recall physical activity questionnaire [14] revealed that all participants were habitually active (i.e., 3–4 days per week of continuous exercise of 30–60 min per session).

### Experimental design

Each participant completed one preliminary and one experimental session. During the preliminary session, body height, mass, and density, as well as VO_2_peak were determined. Body height was determined using a stadiometer (Detecto, model 2391, Webb City, MO, USA), while body mass was measured using a digital high-performance weighing terminal (model CBU150X, Mettler Toledo Inc., Mississauga, ON, Canada). Body surface area was subsequently calculated from the measurements of body height and mass [15]. Body density was measured using the hydrostatic weighing technique, and body fat percentage was calculated using the Siri equation [16]. VO_2_peak was measured during an incremental exercise protocol performed on a cycle ergometer (Corival, Lode B.V., Groningen, Netherlands) which consisted of a 2-min warm-up at 40 W followed by 20 W increments every minute until the participant could no longer maintain a pedaling cadence of at least 60 rpm. For the older females, a 12-lead ECG was monitored throughout the maximal exercise test by a qualified technician to detect any abnormalities in heart activity. If abnormalities were detected, participants were excluded from the study and referred to their physician; however, no abnormalities were detected in the participants screened.

The experimental protocol was performed in a whole-body direct air calorimeter regulated to an ambient temperature of 40°C and 15% RH. An equal number of young and older females performed the experimental protocol in the morning and in the afternoon. Participants consumed a light meal or snack before their arrival (approximately 2 hours before testing) and were asked not to run or bike on their way to the laboratory to avoid any thermal stimuli. Additionally, strenuous activity and alcohol were avoided for 24 hours and caffeine for 12 hours before the experimental session. Participants were instructed to drink ~250 mL of water before going to bed the night before the experimental session as well as in the morning of and within 2 hours of the start of the experimental session. Thereafter, no fluid was ingested.

All participants wore a light pair of athletic shorts, sports bra and sandals. Following the placement of sweat capsules, skin blood flow probe, heart rate monitor and core temperature probe/pill, participants rested for a 30-min baseline period on an upright seated cycle ergometer located in the calorimeter. Baseline rest was followed by three bouts of 30-min cycling exercise (Ex) at increasingly greater rates of metabolic heat production of 250 W (Ex1), 325 W (Ex2), and 400 W (Ex3). Each exercise bout was followed by a 15-min recovery period in the direct calorimeter. The workloads were equivalent to a 35.9 ± 5.5% and 37.9 ± 7.8% for Ex1, 47.1 ± 7.8% and 50.6 ± 10.4% for Ex2, and 58.7 ± 9.6% and 62.9 ± 12.8% for Ex3 of their pre-determined VO_2_peak for the young and older females respectively, or a 36 ± 6 W and 35 ± 7 W for Ex1, 60 ± 5 W and 57 ± 8 W for Ex2 and 80 ± 8 W and 76 ± 9 W for Ex3 external workload for young and older females, respectively.

### Measurements

Whole-body evaporative heat loss and dry heat exchange as well as change in body heat storage were quantified using the modified Snellen direct whole-body air calorimeter. A detailed explanation of how direct calorimetry measures whole-body heat loss and heat storage has been described in a previous publication [17]. Also, a full technical description of the fundamental principles and performance characteristics of the Snellen calorimeter is available [18]. In summary, direct calorimetry measured whole-body evaporative loss and dry heat exchange (radiation, conduction, convection), yielding an accuracy of ±2.3 W for the measurement of whole-body heat loss while indirect calorimetry was used to measure metabolic heat production. Electrochemical gas analyzers located outside of the calorimeter (AMETEK model S-3A/1 and CD 3A, Applied Electrochemistry, Pittsburgh, PA, USA) were used to determine the concentration of expired O_2_ and CO_2_ during experimental sessions and subsequently the respiratory exchange ratio (RER). Using the energy equivalent for the full oxidation of carbohydrates (19.63 kJ per L of O_2_ consumed) and fats (21.13 kJ per L of O_2_ consumed), metabolic heat production can be subsequently calculated [17]. To account for respiratory heat exchange, expired air was recycled back into the calorimeter. The change in body heat storage was subsequently calculated by subtracting the total amount of heat produced and heat dissipated over the experimental protocol. The amount of evaporation required to achieve heat balance was calculated by combining the rates of metabolic heat production and dry heat exchange.

Local sweat production was measured using the ventilated capsule technique. A 3.8 cm^2^ plastic capsule was attached to three skin sites (upper back, chest and forearm) with an adhesive ring and topical skin glue (Collodion HV, Mavidon Medical products, Lake Worth, FL, USA). Compressed dry air was passed through the capsule at a rate of 1.0 L·min^-1^. Water content of the effluent air was measured using high precision dew point mirrors (model 473, RH systems, Albuquerque, NM, USA). Local sweat rate was calculated using the difference in water content between effluent and influent air multiplied by the flow rate and normalized for the skin surface area under the capsule.

Laser-Doppler velocimetry was employed for measuring skin blood flow (PeriFlux System 5000, Main control unit; PF5010 LDPM). A laser-Doppler probe (Perimed integrating probe 413, Järfälla, Sweden) was affixed to the skin on the surface of the left forearm in an area which did not seem overly vascular upon visual inspection and provided stable readings at rest. To measure maximal skin blood flow, the heater housing the laser-Doppler probe was heated to 44°C until maximal skin vasodilation was achieved (~40 min) [19].

Esophageal temperature was measured with a thermocouple temperature probe (Mon-a-therm General Purpose Temperature Probe, Mallinckrodt Medical Inc., St-Louis, MO, USA). The esophageal probe was inserted 40 cm past the nostril entrance while the participants sipped water (100–300 mL) through a straw. Visceral temperature was measured using a telemetric pill (VitalSense ingestible capsule thermometer is a Class II Medical Device according to 21 DFR 8982.1845; Mini Mitter Company Inc.) which moves freely and unobstructed through the digestive tract and is generally eliminated within 48 hours of ingestion [20]. The telemetric pill provides an estimate of internal body temperature. Mean skin temperature was calculated as the weighted average of 4 skin temperature measurements: upper trapezius 30%, chest 30%, quadriceps 20%, and back calf 20% [21]. Data were collected in 15-s intervals and were displayed and recorded in spreadsheet format using a HP Agilent data acquisition module (model 3497A; Agilent Technologies Canada Inc., Mississauga, ON, Canada) and a personal computer with LabVIEW software (Version 7.0, National Instruments, Austin, TX, USA).

Heart rate was monitored, recorded continuously, and stored using a Polar coded WearLink and transmitter, Polar RS400 interface, and Polar ProTrainer 5 software (Polar Electro Oy, Finland).

### Statistical analysis

For all variables, minute averages were calculated to carry out the statistical analyses. Baseline values were obtained by averaging the last 5–10 min of data during the 30-min baseline resting period. Mean body temperature was calculated as: 0.9 × esophageal temperature **+** 0.1 × mean skin temperature [22]. Whole-body evaporative heat loss was plotted against the corresponding mean body temperature. Thereafter, the onset threshold and thermosensitivity of whole-body evaporative heat loss during each exercise period was determined using the linear portion of each response and analyzed using a segmented regression analysis as described by Cheuvront *et al*. (2009) using a computer algorithm (GraphPad Prism 6.0, GraphPad Software, La Jolla, CA, USA) [23]. The onset threshold corresponded to the intercept of the regression line with the evaporative heat loss values at rest, while the thermosensitivity was defined as the slope of the regression line. The time constant (τ, time it takes to reach 63.2% of the total response) and amplitude (difference between evaporative heat loss at the onset and at the end of each exercise bout) of the evaporative heat loss response was calculated for each exercise bout.

Physical characteristics, baseline values and cumulative changes in body heat storage were analyzed using independent samples *t* tests. Dependent variables of rates of metabolic heat production, whole-body evaporative heat loss and dry heat exchange, evaporative requirement for heat loss, changes in body heat storage, as well as esophageal, visceral and mean skin temperatures, local sweat rates and skin blood flow, heart rate responses, evaporative heat loss onset thresholds, thermosensitivities, time constants, and amplitudes were analyzed to compare responses as a function of increasing heat loads (primary analysis). For this purpose, we used a two-way analysis of variance (ANOVA) performed with one factor of age (2 levels: young and older) and the repeated factor of either end exercise (three levels: Ex1, Ex2, Ex3) or end recovery (three levels: Rec1, Rec2, Rec3). We conducted a secondary analysis to further examine whole-body evaporative heat loss by determining at what time point differences in whole-body evaporative heat loss between young and older females occur during each exercise heat load separately. To do so, we used a two-way ANOVA to compare whole-body evaporative heat loss between groups for each heat load separately with a repeated factor of time (six levels: 5, 10, 15 20, 25 and 30 min) and a non-repeated factor of group (two levels: young and older). When a significant main effect was observed, *post hoc* comparisons were carried out using the Bonferroni procedure. The level of significance for all analyses was set at p≤0.05. Statistical analyses were performed using commercially available statistical software (GraphPad Prism 6.0, GraphPad Software, La Jolla, CA, USA). All values are reported as mean ± standard deviation.

## Results

### Responses as a function of increasing heat loads—Whole-body direct calorimetry

#### Baseline and Exercise

There were no differences (p = 0.28) in baseline rates of metabolic heat production between the young (94 ± 14 W) and older (87 ± 12 W) females. By experimental design, the rate of metabolic heat production increased from Ex1 to Ex2, Ex1 to Ex3 and Ex2 to Ex3 in both young and older females (p<0.001), but was similar between age groups for Ex1 (young: 251 ± 7 W; older: 253 ± 17 W), Ex2 (young: 328 ± 7 W; older: 330 ± 6 W) and Ex3 (young: 404 ± 8 W; older: 406 ± 8 W) (p = 0.45). Furthermore, no differences were observed for the rate of dry heat exchange at baseline (young: -65 ± 14 W; older: -62 ± 14 W, *P* = 0.59) or during exercise (p = 0.52) between groups, but did change over time (p = 0.004) such that the rate of dry heat gain was greater at the end of Ex2 compared to Ex1 for the older females (p<0.05). The rates of dry heat exchange at the end of each exercise bout were: young: -79 ± 11 W and older: -75 ± 19 W for Ex1; young: -82 ± 9 W and older: -79 ± 19 W for Ex2 and young: -85 ± 9 W and older: -80 ± 19 W for Ex3. Consequently, the evaporative requirement for heat loss did not differ between age groups at baseline (young: 159 ± 16 W; 149 ± 13 W, p = 0.14) or during exercise (p = 0.78), but did increase from Ex1 to Ex 2, Ex1 to Ex3 and Ex2 to Ex3 (p<0.001). As a result, the net heat load for each exercise bout was 329 ± 24 W (Ex1), 409 ± 17 W (Ex2) and 488 ± 16 W (Ex3).

Whole-body heat loss during exercise was solely due to evaporative heat loss as the negative rate of dry heat exchange resulted in a net dry heat gain. Rates of whole-body evaporative heat loss and the evaporative requirement for heat loss during baseline and exercise are presented in Fig. 1. The rate of evaporative heat loss at baseline was lower in the older compared to young females (young: 115 ± 25 W; older: 88 ± 24 W, p = 0.02). Additionally, despite exercising at similar requirements for heat loss, a main effect of age on the rate of whole-body evaporative heat loss was observed (p = 0.02) such that the rate of evaporative heat loss was greater for the young compared to the older females at the end of Ex2 and Ex3. Furthermore, the rate of evaporative heat loss increased from Ex1 to Ex2, Ex1 to Ex3 and Ex2 to Ex3 in both groups (p<0.001), but was 10.2%, 11.6% and 12.4% lower in the older compared to young females at the end of Ex1, Ex2 and Ex3, respectively.

**Fig 1:** Mean ± standard deviation rates of evaporative heat loss (circles) and the required amount of evaporation for heat balance (E_req_, squares) measured at baseline and over three 30-min exercise bouts (Ex 1, Ex 2 and Ex 3) and three 15-min recovery bouts (Rec 1, Rec 2 and Rec 3) in a hot, dry (40°C, 15% RH) environment in young (grey) and older (white) females. There were no differences in the required amount of evaporation for heat balance between groups. Significant difference (p≤0.05) in evaporative heat loss from young is denoted by an asterisk (*). Significant difference from Ex1/Rec1 is denoted by a cross (†). Significant difference from Ex2/Rec2 is denoted by a double cross (‡).

The changes in body heat storage are presented in Fig. 2. The amount of heat stored in the body increased significantly between each exercise bout in both the young and older females (p<0.001). Additionally, there was a main effect of age on change in body heat storage during exercise (p = 0.002), whereby the young females had a lower amount of heat stored for all three exercise periods (Ex1–3) compared to the older females.

**Fig 2:** Mean ± standard deviation values for changes in body heat storage during each exercise/recovery cycle as well as the total change in body heat storage over the exercise protocols in a hot, dry (40°C, 15% RH) environment. The solid bars represent changes in body heat storage during exercise and the striped bars represent changes in body heat storage during recovery. The grey bars/stripes represent the young group and the white bars/black stripes represent the older group. Significantly different (p≤0.05) from young is denoted by an asterisk (*). Significant difference from Ex1/Rec1 is denoted by a cross (†). Significant difference from Ex2/Rec2 is denoted by a double cross (‡).

#### Recovery

Rates of whole-body evaporative heat loss and the evaporative requirement for heat loss during recovery are presented in Fig. 1. There were no age-related differences in the rate of metabolic heat production during any of the recovery periods (p = 0.18), but the rate of metabolic heat production was significantly lower (p = 0.03) for Rec3 relative to Rec1 and Rec2 in the older females. Furthermore, there was no main effect of age on the rate of whole-body evaporative heat loss (p = 0.55), although evaporative heat loss increased from Rec1 to Rec2 and Rec1 to Rec3 in both young and older females. Moreover, dry heat exchange (p = 0.42) and the evaporative requirement for heat loss (p = 0.48) were similar between age groups at the end of the recovery periods and did not change over time (p>0.05).

The changes in body heat storage during recovery and total heat storage (Ex plus Rec) are presented in Fig. 2. The amount of body heat dissipated (and therefore resulting in a decrease in body heat storage) was significantly greater compared to the previous recovery period in both young and older females (p<0.001) due to the greater amount of heat stored during exercise, but did not differ between age groups during any of the recovery periods (p = 0.79). However, there was a main effect of group on the total body heat storage (p = 0.02), whereby the young females stored significantly less heat by the end of the three exercise/recovery cycles compared to the older females.

### Onset thresholds, thermosensitivities, time constants and amplitudes for whole-body evaporative heat loss

Mean body temperature onset thresholds, thermosensitivities, time constants and amplitudes for whole-body evaporative heat loss during each exercise bout are presented in Table 1. The mean body temperature onset threshold for whole-body evaporative heat loss increased from Ex1 to Ex2 in the older females and from Ex2 to Ex3 in both the young and older females (p<0.001). Moreover, the onset threshold for whole-body evaporative heat loss was significantly different between groups (p = 0.02) such that the onset of evaporative heat loss occurred at a greater mean body temperature for Ex2 and Ex3 for the older females compared to the young females. Also, the thermosensitivity of evaporative heat loss was significantly lower for Ex3 compared to both Ex1 and Ex2 in the older females (p>0.05). However, there was no significant difference in thermosensitivity between age groups (p = 0.10). Furthermore, the time constant for the rate of evaporative heat loss decreased from Ex1 to Ex2 and Ex1 to Ex3 in both young and older females, but was not different between young and older females (p = 0.41) during exercise. In contrast, a main effect of age was evident for the amplitude of evaporative heat loss (p = 0.05) such that the older females had significantly lower amplitudes for Ex2 and Ex3, and increased from Ex1 to Ex2 and Ex1 to Ex3 in the young females only (p<0.05).

**Table 1:** Esophageal, visceral and mean skin temperature responses during each exercise (Ex)/recovery (Rec) cycle and onset thresholds, thermosensitivities, time constants and amplitudes of evaporative heat loss for each exercise bout.

T_es,°_C	Ex1	Rec1	Ex2	Rec2	Ex3	Rec3
**Young**	37.44±0.23	37.33±0.24	37.74±0.32†	37.42±0.19	38.12±0.42† ‡	37.56±0.29†
**Older**	37.59±0.15	37.51±0.20	37.96±0.18†	37.65±0.29	38.33±0.22† ‡	37.91±0.41* † ‡
**T**_**visc,°**_ **C**						
**Young**	37.55±0.26	37.49±0.12	37.94±0.28†	37.77±0.22†	38.17±0.21† ‡	37.85±0.14†
**Older**	37.65±0.28	37.60±0.27	37.90±0.22†	37.76±0.21	38.15±0.31† ‡	38.00±0.35† ‡
**T**_**Sk,°**_ **C**						
**Young**	35.65±0.20	35.59±0.27	35.80±0.28	35.63±0.29	35.92±0.40	35.78±0.33‡
**Older**	35.64±0.28	35.53±0.25	35.76±0.41	35.48±0.33	35.08±0.47† ‡	35.64±0.38‡
**Onset threshold of evaporative heat loss,°C**						
**Young**	36.92±0.30		37.06±0.19		37.20±0.20†	
**Older**	37.04±0.15		37.33±0.19* †		37.50±0.26* † ‡	
**Thermosensitivity of evaporative heat loss, W·°C** ^**-1**^						
**Young**	569±152		495±144		425±220	
**Older**	570±222		392±243		246±146† ‡	
τ, **min**						
**Young**	10.4±2.6		5.0±1.3†		4.9±1.0†	
**Older**	10.6±3.8		7.0±3.3†		4.7±1.9†	
**Amplitude, W**						
**Young**	153±33		191±27†		214±31†	
**Older**	167±24		134±57*		160±70*	

Values are mean ± standard deviation.

T_es_, esophageal temperature.

T_visc_, visceral temperature.

T_Sk_, mean skin temperature.

τ, time constant. Mean body temperature was used to calculated the onset threshold and thermosensitivity.

*Significant difference from young females.

†Significant difference from Ex1/Rec1.

‡Significant difference from Ex2/Rec2.

### Esophageal, visceral mean skin temperatures

#### Baseline and Exercise

Esophageal, visceral and mean skin temperatures during exercise are presented in Table 1. Baseline values for esophageal (young: 37.14 ± 0.26°C; older: 37.18 ± 0.18°C), visceral (young: 37.22 ± 0.25°C; older: 37.25 ± 0.22°C) and mean skin (young: 35.44 ± 0.35°C; older: 35.54 ± 0.26°C) temperatures were similar between groups (all p>0.05). Esophageal and visceral temperature increased between each exercise bout (Ex1 to Ex3) in both the young and older females (p<0.001) while mean skin temperature was greater for Ex2 and Ex3 relative to Ex1 in the young (p = 0.04) for Ex3 relative to Ex1 in the older females (p<0.001). However, there was no main effect of age on esophageal (p = 0.09), visceral (p = 0.89) or mean skin (p = 0.81) temperatures during exercise. Similar findings were observed when core and mean skin temperatures were presented as a change from baseline; that is, there was no main effect of age on esophageal (p = 0.15), visceral (p = 0.91) or mean skin (p = 0.73) temperatures from baseline resting values.

#### Recovery

Recovery values for esophageal, visceral and mean skin temperatures are presented in Table 1. Esophageal and visceral temperatures were significantly greater at the end of Rec3 relative to Rec1 in both young and older females and to Rec2 in the older females only (p<0.001), but mean skin temperature was greater for Rec3 relative to Rec2 in both groups (p<0.001). In addition, there was a main effect of age on esophageal temperature during recovery (p = 0.04), such that the older females had a significantly greater esophageal temperature at the end of Rec3 compared to the young females (p<0.05). In contrast, visceral (p = 0.41) and mean skin (p = 0.40) temperatures were not different between age groups during recovery.

### Local heat loss and heart rate responses

#### Baseline and Exercise

Local sweat rate (chest, back and forearm), local skin blood flow (forearm) and heart rate values are presented in Table 2. There were no differences between groups in local sweat rates during baseline resting for sweat rate measured on the chest (young: 0.14 ± 0.06 mg·min^-1^·cm^-2^; older: 0.14 ± 0.06 mg·min^-1^·cm^-2^, p = 0.98), back (young: 0.20 ± 0.16 mg·min^-1^·cm^-2^; older: 0.19 ± 0.06 mg·min^-1^·cm^-2^, p = 0.78) and forearm (young: 0.16 ± 0.12 mg·min^-1^·cm^-2^; older: 0.13 ± 0.02 mg·min^-1^·cm^-2^, p = 0.36) skin sites. Local sweat rate at all three sites increased significantly from one exercise bout to the next in both the young and older females (p<0.001). On the other hand, sweat rates were similar during exercise between age groups at the chest (p = 0.78), back (p = 0.99) and forearm (p = 0.61) skin sites. Furthermore, local skin blood flow did not differ between age groups at baseline (young: 43.3 ± 17.1%; older: 34.9 ± 21.1%, p = 0.37) or during any of the three exercise bouts (p = 0.28), but did increase from Ex1 to Ex2 in the older females (p = 0.009). Heart rate was significantly greater at the end of Ex2 relative to Ex1 and at the end of Ex3 relative to Ex2 in both the young and older females (p<0.001) but did not differ between age groups during exercise when presented as either absolute (p = 0.07) or as a percentage of maximum (p = 0.80).

**Table 2:** Local heat loss and heart rate responses during each exercise (Ex)/recovery (Rec) cycle.

	Ex1	Rec1	Ex2	Rec2	Ex3	Rec3
**LSR—Chest, mg·min** ^**-1**^ **·cm** ^**-2**^						
**Young**	0.37±0.07	0.20±0.04	0.51±0.12†	0.26±0.09†	0.62±0.15† ‡	0.27±0.11†
**Older**	0.40±0.13	0.22±0.08	0.55±0.17†	0.26±0.12	0.63±0.22† ‡	0.34±0.11† ‡
**LSR—Back, mg·min** ^**-1**^ **·cm** ^**-2**^						
**Young**	0.52±0.27	0.26±0.16	0.69±0.27†	0.31±0.14	0.84±0.40† ‡	0.30±0.11
**Older**	0.54±0.16	0.32±0.10	0.71±0.22†	0.39±0.17	0.82±0.24† ‡	0.47±0.23
**LSR—Arm, mg·min** ^**-1**^ **·cm** ^**-2**^						
**Young**	0.39±0.19	0.19±0.10	0.55±0.19†	0.25±0.13	0.69±0.29† ‡	0.25±0.11
**Older**	0.38±0.13	0.24±0.10	0.53±0.19†	0.25±0.08	0.57±0.21† ‡	0.34±0.13
**SkBF, % of max**						
**Young**	52.1±15.9	43.7±16.4	56.5±13.5	45.3±17.7	57.0±17.3	45.5±16.1
**Older**	57.1±14.2	41.7±20.2	65.1±14.5†	46.2±17.8	65.1±10.6	44.5±21.3
**HR, beats·min** ^**-1**^						
**Young**	117±18	87±17	140±22†	95±18†	161±19† ‡	105±20† ‡
**Older**	103±10	82±8	123±9†	85±9†	146±8† ‡	91±14† ‡
**HR, % of max**						
**Young**	64±9	48±10	77±12†	52±10†	88±10†‡	58±11† ‡
**Older**	64±5	51±4	77±5†	53±6†	91±5† ‡	56±8†

Values are mean ± standard deviation.

LSR, local sweat rate.

SkBF, skin blood flow.

HR, heart rate. % of max, percentage of individual’s maximum.

†Significant difference from Ex1/Rec1.

‡Significant difference from Ex2/Rec2.

#### Recovery

Local sweat rate, skin blood flow and heart rate values during recovery are presented in Table 2. Local sweat rate was greater for Rec2 compared to Rec1 on the chest in the young and greater for Rec3 compared to both Rec1 and Rec2 on the chest and forearm in the older females (p<0.05), but were otherwise stable during recovery. Furthermore, local sweat rates were similar between groups at the chest (p = 0.75), back (p = 0.99) and forearm (p = 0.61) skin sites during recovery. Moreover, no differences in local skin blood flow were measured over recovery time (p>0.05) or between age groups (p = 0.96) during recovery. Heart rate was significantly greater at the end of Rec2 and Rec3 compared to Rec1 in both the young and older females and was also greater at the end of Rec3 compared to Rec2 in the young females (p>0.05), but was not different between age groups during recovery for absolute (p = 0.21) or percentage of maximum (p = 0.81) values.

### Time dependent changes of evaporative heat loss for each heat load

When each heat load was analyzed separately, a main effect of age on rates of whole-body evaporative heat loss was measured for Ex1 (p = 0.05), Ex2 (p = 0.02) and Ex3 (p = 0.009). This was evidenced by the rate of whole-body evaporative heat loss being lower in the older females at 5 and 10 min for Ex1 (p<0.05), which was most likely the result of the lower rate of evaporative heat loss in the older females during baseline. Moreover, the rate of evaporative heat loss was lower in the older females at 20, 25 and 30 min for Ex2 and at 10, 15, 20, 25 and 30 min for Ex3 when compared to young females (p<0.05).

## Discussion

We showed that the maximal rate of whole-body evaporative heat loss achieved during the moderate (Ex2, 325 W) and highest (Ex3, 400 W) heat load employed was significantly lower in older compared to young females matched for aerobic fitness, body surface area and body composition. Furthermore, we showed for the first time that the degree of impairment in evaporative heat loss between the young and older females is greater as the requirement for heat loss increases. Moreover, we showed that the onset threshold for the activation of whole-body evaporative heat loss was delayed in older females relative to their younger counterparts for the second and third heat loads. This was further exacerbated by a significantly more pronounced decrease in the thermosensitivity of the response measured during the successive exercise bouts in the older females. When combined with the attenuated rate of whole-body evaporative heat loss measured throughout the exercise bout, the older females stored significantly more heat than their younger counterparts and the magnitude of increase was more pronounced with increases in the level of heat stress and therefore requirement for heat loss. Of particular note, these impairments in whole-body evaporative heat loss and body heat storage were not paralleled by differences in local heat loss responses of sweating and skin blood flow or increases in core temperature assessed by esophageal and visceral temperature. Finally, no age-related differences in heat loss or heat storage were observed during any of the recovery periods with the exception of esophageal temperature being greater in the older females at the end of the final recovery period.

### Capacity for whole-body evaporative heat loss

Keeping in line with our study hypothesis, we observed that the capacity for whole-body evaporative heat loss was significantly reduced in older compared to young females at the two highest requirements for heat loss (Fig. 1). Although the time constant of the evaporative heat loss response was similar between the young and older females during the exercise bouts, the younger females exhibited greater amplitudes of change in evaporative heat loss for Ex2 and Ex3 (Table 1). Thus, the younger females achieved greater levels of evaporative heat loss within the same amount of time as the older females during Ex2 and Ex3. Impairments in the capacity to dissipate heat in older females have also been reported by Anderson and Kenney [9] who observed a reduction in sudomotor activity in older relative to young females at heat loads similar to that of Ex2 (i.e., exercise at 40% VO_2_peak and ambient conditions of 48°C and 15% RH). In the present study, we observed that older females attained a lower level of evaporative heat loss at the end of the second and third heat load, while no difference was measured at the end of the first heat load which suggests that sudomotor activity is impaired in older females above a heat load threshold equivalent to ~330 W. Furthermore, our exercise model of progressive increases in the evaporative requirement for heat loss allowed us to evaluate if the magnitude of difference in the body’s physiological capacity to dissipate heat becomes greater with progressive increases in heat load. We observed that the separation in the rate of evaporative heat loss between the young and older females was more pronounced with each exercise heat load (Ex1 = 10.2%, Ex2 = 11.6% and Ex3 = 12.4%) despite the same increases in the requirement for heat loss. Altogether, these results suggest that the maximal level of whole-body evaporative heat loss achieved was lower in the older compared to young females for the two highest heat loads employed, and the magnitude of impairment became more pronounced as the heat load increased.

In order to determine whether the age-related impairments in heat loss are due to central and/or peripheral modulations of sudomotor function, the onset threshold and thermosensitivity of whole-body evaporative heat loss can be examined in the context of the observed age-related changes whole-body evaporative heat loss [24]. Previous studies have reported that older adults have an increased mean body temperature threshold for the onset of sweating during heat stress [25,26,27,28]. However, this finding is not always consistent whereby some studies observed no differences in the mean body temperature at which sweating began [12,29,30,31]. As noted earlier, we observed an increase in the onset threshold for evaporative heat loss in the older females for Ex2 and Ex3 (Table 1) which is reflective of the greater heat storage for the older females over time. Furthermore, this was exacerbated by a significant reduction in the thermosensitivity of the response measured between Ex2 and Ex3 in the older females only. Taken together, our findings demonstrate that whole-body sudomotor activity is attenuated with progressive increases in body heat storage in older females. Given that the onset threshold represents a central modulation whereas the thermosensitivity of the response represents a peripheral modulation [24], our findings indicate that the age-related impairments in whole-body sudomotor activity in older females may be attributed to both a central and peripheral modulation of heat loss; a response which we show to be heat load dependent.

### Time-dependent changes in whole-body evaporative heat loss

In addition to comparing the maximal rate of whole-body sudomotor capacity achieved during exercise in older relative to young females, we also assessed the time-dependent changes in whole-body evaporative heat loss for each exercise heat load. Despite observing no significant differences in the maximal level of evaporative heat loss achieved at the end of the first exercise bout between age groups, impairments in whole-body evaporative heat loss were evident during the first 10 min of Ex1, but were similar between groups thereafter. Given that the onset and thermosensitivity for whole-body evaporative heat loss did not differ between groups for Ex1, the lower rate of evaporative heat loss measured for the older females during the early stages of Ex1 was likely due to their lower rate of evaporative heat loss at baseline. In contrast to Ex1, age-related differences in whole-body evaporative heat loss occurred as early as 20 min into Ex2 and 10 min into Ex3 and remained lower for the duration of the 30-min exercise bout. This time dependent decrease in evaporative heat loss can be attributed to a delayed activation of the response in the older females which was paralleled by a progressively greater reduction in thermosensitivity measured during the successive exercise bouts in the older females only. Consequently, the impaired ability to dissipate heat in the older females resulted in a 40%, 57% and 47% greater change in body heat storage compared to young females for Ex1, Ex2 and Ex3, respectively. While Anderson and Kenney [9] reported lower sweat rates after 30 min of exercise at 40% VO_2_peak in a hot, dry environment (48°C, 10% RH) and Larose *et al*. [8] observed a lower rate of whole-body evaporative heat loss in older females as early as 10 min after the onset of exercise at a moderate heat load (i.e., ~320 W), we showed that as the heat load increases, the separation in whole-body evaporative heat loss between young and older females occurs earlier into exercise, thereby causing a greater amount of heat to be stored in the body. Our findings demonstrate that age-related impairments in the physiological capacity to dissipate heat are exacerbated with increases in the level of heat stress, and therefore as the requirement for heat loss becomes greater.

### Core temperature and local heat loss responses

In contrast to the greater heat storage measured for the older females for each exercise bout, differences in esophageal temperature responses were not evident until the very end of the intermittent exercise protocol (end of Rec3) (Table 1). Furthermore, no differences between groups for visceral temperature were observed at any stage of exercise or recovery. Whole-body calorimetry provides an accurate measure of changes in whole-body heat content whereas surrogate measures of body core temperature only represent regional changes in heat content. Regional tissue temperature at any point in time is the result of regional differences in metabolic rate, conductive heat loss to adjacent tissues, and deep and peripheral convective blood flow [17]. Thus, the disparity between body heat storage and core body temperatures can be ascribed to regional variations in tissue blood flow leading to differences in heat transfer/distribution between internal tissues, which occurs to a greater extent in older adults [32]. Of note however, the cumulative amount of heat stored by the end of the exercise-rest protocol was 42% greater in the older compared to young females, which was comparable to the 41% greater increase in esophageal temperature. This was also a similar finding to Larose *et al*. [8] who showed that the cumulative change in body heat storage and net change in rectal temperature were both ~63% greater in older females at the end of the exercise-rest cycles. Thus, despite the differences in heat distribution/storage at the beginning of the Ex/Rec cycles, it appears that core temperature gradually increases to reflect the changes in total body heat storage.

In the present study, we measured whole-body heat loss in parallel with local sweat rates at the chest, upper back and forearm as well as skin blood flow on the forearm. Despite observing marked differences in whole-body evaporative heat loss between young and older females at the end of the second and third exercise bouts, no differences were measured for local heat loss responses at the end of any of the exercise bouts (Table 2). To date, several studies have observed age-related decrements in sweating which occurred at different rates across various regions of the body [29,33,34,35]. Moreover, a high degree of heterogeneity has been observed between different local measurement sites on the body for both sudomotor activity and skin blood flow in adults of a similar age [35,36,37,38]. These previous observations are consistent with our observation that sweat rates measured on the upper back were greater than those measured on the chest and forearm for both the young and older females (Table 2). Likewise, Smith *et al*. [35] also observed higher sweat rates on the back compared to both the arm and abdomen in young and older adults and Inoue *et al*. [29] observed higher sweat rates on the back compared to the thigh in both young and older males during whole-body heating at rest. Furthermore, although we only measured skin blood flow at one site and therefore are unable to make conclusions on regional variations of skin blood flow from our data, skin blood flow has been reported to be lower on the chest and thigh in older compared to young males, with no apparent differences between groups on the forehead [34]. Ultimately, the discrepancy between local and whole-body heat loss responses may lead to inaccurate conclusions regarding the effect that aging can have on the body’s physiological capacity to dissipate heat in both males and females. Whole-body direct calorimetry provides an accurate assessment of the combined response of the 2–4 million sweat glands across the entire surface of the body which can be used to examine differences in the body’s capacity to dissipate heat between groups.

### Postexercise heat loss responses

In the present study, core temperature and body heat storage remained elevated above baseline levels after each exercise bout (Fig. 1 and Table 2), while local and whole-body heat loss responses rapidly declined. This pattern of response has been observed in previous studies in young adults [17,39] and has been attributed to nonthermal factors overriding the thermal control of heat loss during postexercise recovery [17,39]. Furthermore, despite the greater end-exercise heat storage with successive exercise bouts in the older females, the rates of whole-body heat loss, and subsequently changes in body heat storage, during the postexercise recovery periods were similar between the young and older females. In fact, 7%, 47% and 47% of the heat stored during each exercise bout was lost during Rec1, Rec2 and Rec3, respectively in the young females whereas only 6%, 30% and 36% of the heat stored during each exercise bout was lost during Rec1, Rec2 and Rec3, respectively in the older females. As such, it is possible that the level of influence of nonthermal factors on heat loss postexercise may be even greater in older compared to young females due to the greater heat storage at the end of each exercise bout compared to the young females but similar heat loss responses postexercise. Further research is required to establish the actual contribution of thermal and nonthermal mechanisms governing heat loss postexercise in young and older females.

### Considerations

The older females who volunteered for this study were of similar aerobic fitness as the young females. This is consistent with the studies by Anderson and Kenney [9] and Larose *et al*. [8] who also observed impaired heat loss in older relative to young females of similar aerobic capacity [8,9]. Thus, the decrements in local and/or whole-body heat loss in older females appears to be unrelated to aerobic capacity, but instead may reflect alterations in central and/or peripheral control of sweating associated with advanced aging. It is important to consider that the similar VO_2_peak values between groups in the present study, and others, may indicate that the older females were more physically active than the average older female. In fact, the older females in our study were in the 80 to 90^th^ percentile while the younger females were in the 70 to 80^th^ percentile for aerobic capacity. Since high levels of aerobic fitness associated with regular endurance-type exercise, can improve thermoregulatory control during exercise [40,41,42,43,44], less aerobically fit older females may have an even further attenuated capacity to dissipate heat compared to both young and older, habitually active females.

Given that whole-body heat loss responses between groups were compared using a progressive increase in the exercise-induced heat load, it remains unclear if the pattern and/or magnitude of difference in whole-body heat loss, and therefore body heat storage, observed between groups would differ had each exercise condition been performed on separate days. It is known that there is a greater activation of whole-body evaporative heat loss response following an initial exercise bout, termed the priming effect, and this response occurs irrespective of the age of the individual [3,8]. While we cannot determine how the prior exercise bout might have affected the rate of whole-body evaporative heat loss, and therefore the magnitude of difference in body heat storage between groups, we consistently observed an attenuated rate of heat dissipation in older females relative to their young counterparts irrespective the greater thermal drive associated with the successively greater exercise-induced heat loads. Future studies are required to determine how a prior exercise bout might influence the extent to which these age-related impairments may attenuate whole-body evaporative heat loss, and therefore body heat storage, when exercise is performed at the higher exercise-induced loads where we show the greatest differences between groups to occur.

Finally, another point to consider is that reproductive hormones may influence the thermoregulatory system, whereby estrogen and progesterone levels are reported to alter baseline core temperatures [45,46]. In the present study, two of the older females were on hormone replacement therapy (HRT). There were no significant differences in baseline esophageal temperature between the young females (37.14 ± 0.26°C, n = 10) and older females not on HRT (37.15 ± 0.16°C, n = 8). However, those who were taking HRT had a slightly elevated esophageal temperature (37.32 ± 0.21°C, n = 2). Despite the elevated core temperature at baseline, there were no differences in changes in esophageal temperature (older no HRT: 37.90 ± 0.43°C vs. HRT: 37.96 ± 0.44°C) or body heat storage (older no HRT: 430 ± 174 kJ vs. HRT: 418 ± 10 kJ) between females who were taking or not taking HRT by the end of the exercise/recovery protocol (p>0.05). Furthermore, these values are in sharp contrast to younger females whose change in body heat storage was 247 ± 155 kJ. Thus, HRT did not appear to affect the clear age-related impairments in whole-body heat dissipation causing greater amounts of heat stored in the body of the older compared to young females. Nevertheless, further studies are warranted to fully examine the effects of HRT on whole-body heat storage.

### Summary

We showed that older females demonstrated a lower capacity for whole-body evaporative heat loss compared to young females when exercising in the heat at a rate of metabolic heat production of ≥325 W. Further, we observed a greater separation between age groups with progressive increases in the requirements for heat loss. These increasingly greater impairments in whole-body sudomotor capacity between young and older females were the result of a greater onset threshold and gradual decrease in thermosensitvity for the older females. Ultimately, the impaired capacity to dissipate heat led to greater heat storage in older females which was more pronounced with increases in the level of heat stress.

## Supporting Information

S1 Dataset (XLS)

S2 Dataset (XLSX)
